# Aloe-Emodin Suppresses Oxidative Stress and Inflammation via a PI3K-Dependent Mechanism in a Murine Model of Sepsis

**DOI:** 10.1155/2022/9697887

**Published:** 2022-08-08

**Authors:** Huijie Gao, Yan Ren, Chao Liu

**Affiliations:** College of Pharmacy, Jining Medical University, Rizhao, Shandong, China

## Abstract

**Background:**

This study was designed to assess the impact of aloe-emodin (AE) on oxidative stress and inflammation in a murine model of LPS-induced sepsis. In addition, the mechanistic basis for anti-inflammatory and antioxidant activity was assessed.

**Methods:**

Male ICR mice received an intraperitoneal injection of LPS (10 mg/kg), and the preventive properties of AE (80 or 150 mg/kg) on these mice were assessed by monitoring spleen index, and levels of inflammatory and oxidative stress-related factors. Peripheral blood TNF-*α* and IL-6 levels were assessed via ELISA kits, while changes in hepatic SOD and GSH-Px levels were assessed using appropriate biochemical kits. Splenic PI3K, AKT, and mTOR levels were assessed via qPCR and western blotting.

**Results:**

Relative to animals in the LPS model group, those in the AE treatment groups exhibited reduced spleen index, decreased inflammatory cytokine levels, and improved SOD and GSH-Px activity in liver tissues. Splenic PI3K, Akt, and mTOR levels were also reduced in response to AE treatment.

**Conclusions:**

These findings indicated that AE can alleviate sepsis-related tissue damage, inflammation, and oxidative stress, at least in part by suppressing the PI3K/Akt/mTOR signaling pathway. These results offer a clinical basis for the use of AE to treat sepsis and associated diseases.

## 1. Introduction

Sepsis is a complex condition of severe multiple organ dysfunction caused by a dysfunctional response of the host to infection [1, 2]. Although there have been significant advances in early diagnosis and management for patients suffering from sepsis, effective drugs capable of treating this condition are yet to be established and the disease is still the leading cause of death in intensive care units [3, 4]. Therefore, sepsis remains a major public health problem worldwide. From a mechanistic perspective, sepsis is primarily characterized by excessive inflammation response and unrestrained oxidative stress [5, 6], resulting in severe inflammatory tissue damage driven by TNF-*α*, IL-6, and other proinflammatory cytokines [7, 8].

Lipopolysaccharide (LPS), which is known as endotoxin is a normal component derived from Gram-negative bacteria [9], LPS is highly immunogenic and is involved in the pathogenesis of sepsis, which can lead to “cytokine storm,” intensified oxidative stress, and so on. LPS bind to toll-like receptor 4 (TLR4) in macrophages and triggers downstream signaling cascades as well as the expression of proinflammatory mediators and ROS. High levels of proinflammatory mediators and ROS can lead to a complex condition of severe multiple organ dysfunction known as sepsis [10–12].

Aloe-emodin (AE, 1,8-dihydroxy-3-hydroxymethyl anthraquinone, C_15_H_10_O_5_, Figure 1) is a natural anthraquinone compound, which is mainly derived from dried roots and rhizomes of Chinese medicinal herbs [13], such as *Rheum rhabarbarum* and *Aloe vera*, that are used as traditional medicines in many countries [14–16]. In recent years, numerous pharmacological and clinical studies have identified various therapeutic efficacies of rhubarb, including antibacterial [17], antioxidant [18], anticancer [15], anti-inflammation [19, 20], and other effects. The main active components of rhubarb are anthraquinone derivatives, including emodin, aloe-emodin, rhein, and so on [21]. Emodin and rhein exert anti-inflammatory effects by blocking MAPK and PI3K pathway signaling [22, 23] and antioxidation effects by inhibiting the activation of NF-*κ*B and iNOS expression [24].

Hu et al. demonstrated that aloe-emodin was the bioactive component of rhubarb that confers an anti-inflammatory effect by suppressing the production of NO, interleukin-6 (IL-6), and interleukin-1*β* (IL-1*β*) in LPS-induced RAW264.7 macrophages via inhibition of NF-*κ*B, MAPK, and PI3K pathways [9]. Therefore, aloe-emodin is expected to be an effective treatment for sepsis. In the present study, mice were intragastrically administered AE in order to evaluate the mechanistic basis for its anti-inflammatory and antioxidant activity in a murine model of LPS-induced sepsis as a means of exploring the preventive properties of this natural compound.

## 2. Materials and Methods

### 2.1. Animals

Male ICR mice (6–8 weeks old, 20–25 g, SPF grade) were purchased from Ji'nan Peng Yue experimental animal breeding company (China). Mice were housed in a climate-controlled (22–24°C) SPF facility with free food and water access. All experiments were conducted in accordance with the guidelines of the Chinese Council on Animal Care and were approved by the Animal Care and Use Committee of Jining Medical University (2019-YX-008, Jining, China).

### 2.2. Chemicals and Reagents

AE (C15H10O5, A111278) was from Aladdin Biochemical Technology (Shanghai, China). LPS (*Escherichia coli* 055:B5) and mouse TNF-alpha and IL-6 ELISA kits (Lot. no.20190306) were from Solarbio (Beijing, China). SOD (A001-3-2) and GSH-Px (A005-1-2) test kits were from Jiancheng Bioengineering Institute, Nanjing, China. A PrimeScript RT Master Mix Kit was from TaKaRa (Otsu, Shiga, Japan), while AceQ® qPCR SYBR Green Master Mix (Q111-02) was from Vazyme Biotech (Nanjing, China). Primary antibodies in this study were specific for *α*-tubulin (AT819, Beyotime, China) and PI3K P110 (20584-1-AP, Proteintech, China). Secondary HRP-labeled goat anti-mouse (A0216, Beyotime) and HRP-labeled goat anti-rabbit (A0208, Beyotime) antibodies were also used.

### 2.3. Experimental Model

In total, 40 mice were randomized into five groups: a control group, an LPS model group, a dexamethasone (Dexa) positive control group administered 10 mg/kg Dexa, a low-dose AE group (80 mg/kg), and a high-dose AE group (150 mg/kg). Mice were allowed to acclimate to the laboratory setting for 7 days before experimentation. Animals in the low- and high-dose AE groups were intragastrically administered appropriate doses of AE for 10 days, while mice in the Dexa group were administered Dexa (10 mg/kg) during this time period. Mice in LPS and control groups were administered saline. One hour following compound administration on day 10, mice in the control group were intraperitoneally injected with normal saline, whereas all other mice were injected with LPS (10 mg/kg) to establish the sepsis model. The survival of these mice was then monitored, and mice were sacrificed with pentobarbital sodium 7 hours post-LPS administration to evaluate their weight, blood biochemistry, and spleen/liver status.

### 2.4. Spleen Index Calculation

The spleen index for each mouse was determined as follows: spleen index = spleen weight (mg)/body weight (g).

### 2.5. IL-6 and TNF-*α* Assays

Peripheral blood IL-6 and TNF-*α* levels were assessed using ELISA kits based on provided protocols, with final concentrations being determined by measuring optical density values at 450 nm with a multifunction plate reader.

### 2.6. SOD and GSH-Px Determination

Samples of murine liver tissue (0.5 g) were washed with saline and used to prepare 10% tissue homogenates according to the manual. The activity of GSH-Px and SOD was then measured with appropriate commercial kits based on provided instructions, with respective optical density values of 550 nm (GSH-Px) and 412 nm (SOD) as analyzed with a multifunction plate reader.

### 2.7. qPCR

Trizol was used to extract total RNA from spleen samples based on provided instructions, after which the PrimeScript RT Master Mix was used to prepare cDNA, and SYBR Green Master Mix was used for qPCR analyses. All the primer sequences are listed in Table 1. The 2^−ΔΔCt^ method was used to assess relative gene expression.

### 2.8. Western Blotting

Samples of murine spleen homogenates were lysed using RIPA buffer containing 1 mmol/L PMSF and protease inhibitor cocktail, and protein-containing supernatants were collected. Supernatants were then separated via 10% SDS-PAGE and transferred to PVDF membranes that were blocked using Quick Blocking Buffer and probed overnight with anti-PI3K (1 : 1000) and anti-*α*-tubulin (1 : 2000) at 4°C. Blots were then probed for 2 h with appropriate HRP-linked secondary antibodies, after which an ECL reagent was used for protein band detection.

### 2.9. Statistical Analysis

Data were given as means ± SD and were compared via Student's *t*-tests or one-way ANOVA with Tukey's post hoc test as appropriate. SPSS v18.0 was used for all statistical analyses, with *p* < 0.05 as the significance threshold. All experiments were conducted in triplicate.

## 3. Results

### 3.1. The Impact of AE on Sepsis-Induced Changes in Spleen Index Values

The impact of AE treatment on sepsis was first evaluated by comparing index values in all experiment groups. We found that LPS model mice had significantly higher spleen index values relative to control animals, consistent with successful models. Spleen index values in the Dexa group were significantly lower relative to the LPS group, as were values in the high-dose and low-dose AE groups (Figure 2). As such, AE treatment may be sufficient to alleviate inflammation and associated changes in spleen weight in sepsis model mice.

### 3.2. AE Treatment Suppresses Sepsis-Associated Inflammatory Cytokines Production

We next evaluated the impact of AE on inflammation in our experimental model system by measuring serum inflammatory cytokine levels. We found that LPS treatment was associated with significant increases in TNF-*α* and IL-6 levels relative to control mice (Figure 3, Figure 4). TNF-*α* and IL-6 levels were significantly lower in the Dexa group animals relative to those in the LPS group. In addition, serum TNF-*α* and IL-6 levels were decreased in the high-dose AE groups in a dose-dependent manner relative to the LPS group. These data thus demonstrated that pretreatment with AE is an effective means of suppressing inflammation in sepsis model mice.

### 3.3. Changes in Hepatic SOD and GSH-Px

To evaluate the impact of AE on sepsis, we next assessed hepatic SOD and GSH-Px activity levels in treated mice, as these are important markers of oxidative stress. Relative to control and Dexa group animals, those in the LPS group exhibited marked reduction in SOD and GSH-Px activity, whereas these antioxidant enzyme activities were significantly increased in both AE treatment groups relative to the LPS group (Figure 4). As such, AE was able to effectively decrease oxidative damage in treated sepsis model mice.

### 3.4. AE Treatment Suppresses PI3K-Akt-mTOR Pathway Activation in Sepsis Model Mice

To assess the impact of AE on splenic PI3K-Akt-mTOR pathway activation, we next assessed the expression of pathway-related genes via qPCR and western blotting. LPS model animals exhibited significant increases in PI3K, AKT, and mTOR levels relative to controls (Figure 5), consistent with LPS-induced PI3K-Akt-mTOR pathway activation. Importantly, high- and low-dose AE treatment significantly decreased the expression of all three of these genes in treated animals relative to the LPS model group, indicating that AE can suppress the activation of the PI3K-Akt-mTOR pathway in a murine sepsis model.

## 4. Discussion

Sepsis represents a leading cause of mortality and serious illness among hospitalized patients, and can often lead to fatal multiorgan dysfunction as a result of an inappropriately robust immune response to pathogens that leads to disseminated inflammation [24, 25]. In the past decade, sepsis rates have risen by 30% [26]. Numerous studies have demonstrated the key role of immune dysfunction in the pathogenesis of sepsis [27, 28]. Early deaths from sepsis are typically the result of an overwhelming proinflammatory response, leading to a cytokine storm with multiorgan failure [29].

As the largest peripheral lymphoid organ, the spleen is an important base for various immune cells to live, proliferate, differentiate, conduct immune responses, and produce immune effector substances [30]. Due to its high concentrations of macrophages and extremely rich blood supply, the spleen is very sensitive to LPS, which is considered to be the primary driver of the systemic inflammatory response to sepsis [31–33]. The main cellular targets for LPS are macrophages in the spleen, and LPS binds to toll-like receptor 4 (TLR4) in macrophages and triggers downstream signaling cascades as well as expression of proinflammatory mediators such as TNF-*α* and IL-6 [34, 35]. These factors then drive systemic inflammation and associated septicemic pathology, with IL-6 in particular being an important driver of this response, while TNF-*α* additionally regulates immune cells and is produced in large quantities in the context of sepsis. After the initiation of inflammation, the spleen is congested and massive inflammatory cells proliferate, leading to abnormal enlargement of the spleen. Herein, we found that AE was able to alleviate associated changes in spleen index and suppress LPS-induced TNF-*α*, and IL-6 production, suggesting that it plays an important protective role as an anti-inflammatory agent in our murine sepsis model.

In addition to inflammation, oxidative stress is thought to be a key driver of the pathology of sepsis [36, 37]. Inflammation can increase peroxide levels via driving such oxidative stress [38], and while tissue damage severity in the context of sepsis is correlated with TNF-*α* levels, it is also linked to oxidative damage [39]. SOD and GSH-Px are key antioxidants that counteract such stress [40, 41]. GSH-Px has been shown to protect against inflammation-induced damage in pulmonary tissues [42]. Sepsis is associated with the impairment of the antioxidant defence system, and septicemic model animals exhibit decreased GSH-Px activity in hepatic and renal tissues [43]. In line with this, we found that AE treatment was sufficient to reverse LPS-induced decreases in hepatic SOD and GSH-Px activity of treated mice, consistent with the ability of AE to protect against septic tissue damage by attenuating excessive oxidative stress.

The PI3K/Akt signaling pathway serves to regulate cellular apoptosis, survival, inflammation, and proliferation [44], and is composed of a series of evolutionarily conserved enzymes amenable to targeting with inhibitors of AKT, mTOR, PI3K, and related subunits thereof [45, 46]. Cytokine, hormone, and growth factor signaling almost invariably induce PI3K activation [47]. Such PI3K/Akt signaling has recently been shown to be a core regulator of inflammatory responses [48], and inhibiting this pathway has been shown to effectively suppress inflammatory TNF-*α* and IL-6 production [49]. Herein, we assessed the role of this PI3K/Akt/mTOR pathway in the context of our murine sepsis model, revealing that AE treatment was sufficient to suppress LPS-induced upregulation of PI3K, Akt, and mTOR, thus indicating that this compound inhibited sepsis-related activation of PI3K signaling. Endothelial cell-derived reactive oxygen species (ROS) can also induce PI3K/Akt pathway activation. We found that AE treatment suppressed both inflammatory cytokine production and oxidative stress in LPS-treated mice, while simultaneously suppressing PI3K pathway-related gene expression. As such, our data suggested that AE can attenuate inflammation and oxidative stress by inhibiting this PI3K/Akt/mTOR pathway. The association between AE and the PI3K signaling pathway remains to be clarified in future studies. In summary, we identified AE as a potent anti-inflammatory and antioxidant compound that was able to protect against LPS-induced inflammation in our murine sepsis model at least in part via suppressing PI3K/Akt/mTOR signaling.

Overall, our data highlight a novel mechanism whereby AE can protect against LPS-induced septicemia. These results may guide the design of future therapeutic strategies and suggest that AE warrants further clinical study as a tool for the prevention and treatment of sepsis.

## Figures and Tables

**Figure 1:** Molecular structure of aloe-emodin.

**Figure 2:** Effect of aloe-emodin on spleen index in LPS-induced sepsis in mice. ns, *P* > 0.05, ^*∗∗∗*^*P* < 0.001, ^*∗∗∗∗*^*P* < 0.0001.

**Figure 3:** Effect of aloe-emodin on TNF-*α* (a) and IL-6 (b) levels of mice. ns, *P* > 0.05, ^*∗*^*P* < 0.05, ^*∗∗*^*P* < 0.01, ^*∗∗∗*^*P* < 0.001, ^*∗∗∗∗*^*P* < 0.0001.

**Figure 4:** Effect of aloe-emodin on hepatic SOD (a) and GSH-Px activity (b) levels. ^*∗*^*P* < 0.05, ^*∗∗*^*P* < 0.01, ^*∗∗∗*^*P* < 0.001, ^*∗∗∗∗*^*P* < 0.0001.

**Figure 5:** Effect of aloe-emodin on splenic PI3K, AKT, and mTOR relative expression levels via qPCR (a–c) and western blotting (d). ^*∗∗∗∗*^*P* < 0.0001.

**Table 1:** qPCR primers used in the present study.

Gene	Primer Sequences	
PI3K	Forward	CGAGAGTGTCGTCACAGTGTC
	Reverse	CGAGAGTGTCGTCACAGTGTC

AKT	Forward	ATGAACGACGTAGCCATTGTG
	Reverse	TTGTAGCCAATAAAGGTGCCAT

mTOR	Forward	CAGTTCGCCAGTGGACTGAAG
	Reverse	GCTGGTCATAGAAGCGAGTAGAC

GAPDH	Forward	AACGACCCCTTCATTGAC
	Reverse	TCCACGACATACTCAGCAC

## Data Availability

The figure data used to support the findings of this study are available from the first author upon request.
